# Research on Classification Method of Medical Ultrasound Image Processing Based on Neural Network

**DOI:** 10.1155/2022/8912566

**Published:** 2022-11-23

**Authors:** Fen Gu, Mei Deng, Xi Chen, Li An, Zhen Zhao

**Affiliations:** ^1^Department of Ultrasound, Xijing Hospital, Fourth Military Medical University, Xi'an 710032, China; ^2^Department of Ultrasound, Yuncheng Central Hospital, Shanxi Medical University, Yuncheng 044000, China; ^3^State Key Laboratory for Manufacturing Systems Engineering, Mechanics Institute, Xi'an Jiaotong University, Xi'an 710049, China

## Abstract

In clinical applications, the classification of ultrasound images needs to be processed as an aid to diagnosis. Based on this, a hybrid model of cascaded deep convolutional neural network consisting of two different CNNs and a new classification method are designed and evaluated for its feasibility and effectiveness in ultrasound image classification. A total of 1000 pathological slides of patients with thyroid nodular lesions kept in the Department of Pathology of the First Affiliated Hospital of Lanzhou University, China, were retrospectively collected. After image acquisition, the images were randomly divided into training set, validation set, and test set in the ratio of 4 : 3 : 3. Three convolutional neural network models (VGG 19 model, Inception V3 model, and DenseNet 161 model) with pretraining parameters acquired on the training set were trained, and the models were combined to construct an integrated learning model, and the performance of the models in recognizing pathological images was evaluated based on the test set data. The experimental results show that the VGG 19 model is less effective in classification, with a correct rate of 88.20%, which is lower than that of Inception V3 and DenseNet161 models (92.87% and 92.95%). InceptionV3 and DenseNet161 models have significant advantages in terms of accuracy, number of parameters, and training efficiency, where the DenseNet161 model has faster convergence and better generalization performance, but occupies more video memory in the operation; moreover, the DenseNet161 operation time (1986.48 s) and response time (16 s) are better than the other two models. In addition, the integrated learning of InceptionV3 and DenseNet161 can improve the recognition of pathological images by a single model. Compared with other methods, the performance of the cascaded CNNs proposed in this study is significantly improved, and the multiview strategy can improve the performance of cascaded CNNs. The experimental results demonstrate the potential clinical application of cascaded CNNs, which can provide physicians with an objective second opinion and reduce their heavy workload, in addition to making the diagnosis of thyroid nodules easy and reproducible for people without medical expertise.

## 1. Preface

With the continuous development of society and substantial progress in technology, health issues are receiving more and more attention, which has prompted the development of medical diagnostic techniques in a more advanced direction [1–3]. As an important part of the medical diagnostic field, medical imaging has gradually developed into a relatively independent discipline. In recent decades, medical imaging has developed very rapidly in the field of medical diagnostic technology, and it is an important basis for clinicians to observe, analyze, diagnose, and treat lesions. Medical imaging makes it possible for clinicians to observe lesion sites inside the human body more directly and clearly and to diagnose and treat diseases more accurately [4–6]. With the advent of the digital era, a variety of medical imaging techniques have emerged in medical imaging, such as computed tomography, magnetic resonance imaging, and ultrasound imaging, and these imaging techniques have been widely used in medical diagnosis.

In the field of medical imaging technology, medical ultrasound imaging technology is the most widely used. Medical ultrasound imaging technology combines multiple frontier technologies such as ultrasound physics, biomedicine, and modern electronic detection technology and is a living force in the wave-breaking trend of science and technology. Medical ultrasound diagnosis is the technique of applying ultrasound imaging equipment to the human body to detect tissues and organs and determine whether they are diseased or not [7]. Compared with the clinical applications of computed tomography, X-ray scanning, and magnetic resonance imaging, medical ultrasound diagnostic technology has its unique advantages. First, the propagation and detection medium used in the medical ultrasound imaging technology is ultrasound. Ultrasound has the advantages of high frequency, short wavelength, concentrated energy, good directionality, and strong penetrating power [8]. Second, ultrasound is safe and noninvasive. When the patient is exposed to ultrasound with standard energy, medical ultrasound imaging equipment can achieve safety and noninvasiveness to the human body parts [9]. Third, ultrasound has no radiation to the human body and is safer than the use of X-rays, computed tomography, and MRI [10]. Fourth, medical ultrasound imaging is fast and real time. In contrast, X-rays, computed tomography, and MRI take longer to acquire data, and imaging is slower [11]. Fifth, medical ultrasound imaging equipment is simple and low cost, and with the increasing development of integration technology and digital technology, medical ultrasound imaging equipment is becoming smaller and more integrated, which is very convenient to carry and operate and easy to promote the use [12]. Therefore, more and more ultrasound diagnostic devices have been used in medical diagnosis. It has made a very great contribution to the development and breakthrough of technology in the medical field. Nowadays, medical ultrasound diagnostic equipment has become an indispensable tool in medical diagnosis.

Meraj et al. [13] focused on segmentation of breast lesions by a quantization-assisted U-Net approach, where quantization-assisted U-Net based segmentation in order to isolate the exact lesion region from the ultrasound image. The independent component analysis (ICA) method then uses the separated lesion regions to extract features, which are then fused with deep automatic features. This method has a higher performance compared to the current state-of-the-art variants. However, the disadvantages are insufficient dataset, lack of training for segmentation and classification, and lack of deep learning means for segmentation training. Jabeen et al. [14], on the contrary, are an automated system for breast cancer classification using ultrasound images. The breast ultrasound data were first augmented and then retrained using the DarkNet-53 deep learning model. Features are then extracted from the pooling layer and then the best features are selected using two different optimization algorithms. The selected features were finally fused using the proposed method and subsequently classified using a machine learning algorithm. This method achieves an accuracy of 99.1%. However, this method also has an insufficient number of databases and also lacks a CNN model for breast tumor classification, which is not sufficiently convincing to support the data for breast tumor classification. Irfan et al. [15] used a deep neural network DenseNet201 with migration learning to further validate and secure features rich in target intensity by using transfer learning-based feature extraction. The accuracy of the CNN-activated feature vector and the DenseNet201-activated feature vector combined with the support vector machine (SVM) classifier was 90.11% and 98.45%, respectively. The accuracy of the fused version of feature vector with SVM is 98.9%, which exceeds the other algorithms. However, the limitation of the proposed method is that the feature selection technique was not used. Savelonas et al. [16] used K-nearest neighbor (KNN) and support vector machine (SVM) classifiers for the detection of thyroid nodules with boundary features (compactness, fractal dimension, and local echogenic differences), and the best result of SVM was an AUC of 0.95. Iakovidis et al. [17] used local binary patterns (LBP), fuzzy local binary patterns (FLBP), and fuzzy grayscale histogram (FGLH) to train SVM with a polynomial kernel for thyroid nodule detection. The best performance was estimated to be 97.5% according to AUC. Keramidas et al. [18] also used SVM and KNN classifiers to detect thyroid nodules based on the features of FLBP and FGLH. Their best classification accuracy was estimated to be more than 95%. Bibicu et al. [19] extracted first-order statistical features (mean, standard deviation, skewness, kurtosis, energy, and entropy) to detect thyroid nodules by *Z* or the *t*-statistic test. It was able to identify thyroid nodules with a correct classification rate of 83% when analyzing the whole image and 91% when analyzing the ROI. Although these studies obtained encouraging results, they were mostly based on a series of preprocessing based on hand-designed features extracted from the images. Moreover, the extraction of effective features is a challenging task that requires the help of classifiers for the latter steps of feature selection and feature integration.

To overcome the above difficulties, this study proposes to classify the benign and malignant of common pathology-thyroid nodular disease by using ultrasound image imaging histology and detecting thyroid nodules from two-dimensional ultrasound images using cascaded convolutional neural networks (CNNs). CNN is a deep learning model, and the main structure of CNN includes convolutional layer, pooling layer, and fully connected layer. The convolution layer can learn image features from the input image in the form of a local matrix through convolution operations while preserving the spatial relationship between pixels so that only some nodes between adjacent connected layers need to be connected, i.e., locally connected. The pooling layer can gradually reduce the spatial scale of the input representation, i.e., reduce the feature tensor dimension, simplify operations, reduce the time and space complexity of the network, and avoid overfitting, while being able to reduce the network's sensitivity to irrelevant changes, redundant errors, and small transformations in the input image, allowing more neuron nodes to flow to the main features, thus improving the robustness of the features and speeding up the acquisition of key features. The fully connected layer plays the role of mapping the features acquired by the network during training to the sample labeling space. Each neuron in the fully connected layer is fully connected to all neurons in its previous layer, which can integrate local information with category differentiation in the convolutional and pooling layers.

In this study, our cascaded CNN takes image patches of thyroid nodules and normal thyroid as input and then generates feature maps as output. Multiple intermediate layers apply convolution, pooling, and normalization operations to transform the input into the output. The network contains millions of trainable parameters that are tuned on a set of manually delineated thyroid image data. In addition, the CNN automatically learns a hierarchy of effective features from the thyroid ultrasound images by building high-level features from low-level features. First, the region of interest (i.e., thyroid nodule region) of the ultrasound image is roughly delineated by the physician. Second, a CNN (with 15 convolutional layers and 2 ensemble layers) is trained to segment the thyroid nodules and generate the corresponding segmentation probability maps. Third, all segmentation probability maps are partitioned into different connected regions by a new segmentation method, which consists of successive binarization operators, erosion operators, and dilation operators. Finally, another CNN (with four convolutional and four pooling layers) is used to detect thyroid nodules based on ultrasound image patches relabeled by the segmentation probability map. The main contributions of this study include the following three aspects:

1. Cascaded CNNs are able to compress image features, discard redundancy, effectively reduce the number of parameters in the neural network, and improve network learning efficiency compared to traditional neural networks, which are suitable for processing complex and large 2D ultrasound images for detecting medical images of thyroid nodules.
2. A hybrid method based on CNNs is developed to detect thyroid nodules, which is a cascade method based on a special segmentation method, and two different CNN architectures with different convolutional layers, pooling layers, fully connected layers, etc. In addition, a multiview strategy is used to improve the performance of cascaded CNNs.
3. The cascaded CNNs proposed in this study can automatically extract and select effective features from thyroid images without any complex preprocessing. Compared with other conventional methods, the method of cascaded CNNs can significantly improve the detection of thyroid nodules. In addition, effective preprocessing and data enhancement strategies for thyroid ultrasound images can improve the diagnostic performance.

## 2. Research Methods

The research methods included in this study are described in the following sections.

### 2.1. Instrumentation

Instrumentation includes KJ-2V5M type color ultrasound (Nanjing Keyue Medical Equipment Co., Ltd.), DW-T6 type color ultrasound (Jinan Alaibao Instruments and Equipment Co., Ltd.), and KR-S80 type color ultrasound (Xuzhou Kyle Medical Instruments Co., Ltd.).

### 2.2. Image Acquisition

In this study, 400 patients with thyroid nodular lesions, 500 males and 500 females, with an average age of (45.8 ± 10.5) years, of whom 665 were benign nodules and 335 were malignant nodules, were selected and characterized by examination in the ultrasound room of the Department of Functional Examination of the First Affiliated Hospital of Lanzhou University. All patients were scanned on their affected areas using ultrasound KJ-2V5M, DW-T6, or KR-S80 ultrasonography machines, respectively. All collected cases underwent surgery for thyroid nodules, and pathological test results were used as criteria for benign and malignant diagnosis.

### 2.3. Software and Hardware Tools

#### 2.3.1. Software Tools

1. The subject uses Python 3.7 as the development language. Python as a computer programming language is powerful, lightweight, convenient, mature, and stable. Compared to other programming languages, the Python language has a large selection of frameworks and rich-class libraries for neural network model training and has significant advantages such as easy development, low-code volume, and low cost of using internal types and library functions' advantages [20]. Matlab R2021a was also used as an auxiliary software tool to implement some of the arithmetic, testing, tabulation, and preprocessing tasks.
2. The computing component uses NVIDIA's unified computing device architecture technology, the universal parallel computing architecture, which incorporates the CUDA instruction set architecture (ISA) and the GPU's internal parallel computing engine. The computational power of the GPU, the graphics processing unit, is leveraged to address the complex and large computational volumes in deep learning.
3. The deep learning framework uses the Pytorch framework developed by Facebook in Python on the basis of the deep learning framework Torch, which is rich in features and has many APIs, and can quickly complete the construction and training of deep neural network models. Compared to the TensorFlow framework, the dynamic nature of the Pytorch framework makes the training process and changes in data more intuitive, and the process of calculating and modifying weights more convenient.

#### 2.3.2. Hardware Tools

The hardware part uses a computer equipped with Windows 10 version, the CPU is i9-12900K, 16 cores, and 24 threads processor and the main frequency is 3.1 GHz. The GPU is NVIDIA GeForce GTX3070Ti.

### 2.4. Cascaded CNN Architecture

In this study, we designed a cascaded CNN-based model containing two CNN architectures and a segmentation method for detecting thyroid nodules from ultrasound images.  Figure 1 and Tables 1 and 2 show the detailed structure of the CNNs, respectively. The first CNN (referred to as CNN15) architecture consists of 15 convolutional layers and 2 pooling layers. The output of the previous layer is used as the input of the current layer. All feature mappings generated in the current layer are connected to all feature mappings in the previous layer by convolutional filters.

The first convolutional layer has a filter size of 13 × 13, a step size of 2 pixels, and a fill size of 6 pixels, generating 96 feature maps of size 177 × 177. The next two convolutional layers both generate 256 feature maps of size 45 × 45 by a filter of size 5 × 5. In the second convolutional layer, the fill size is 2 pixels and the step size is 2 pixels. In the second convolutional layer, a 2-pixel fill and a 1-pixel step size are used. In the third convolutional layer, a fill of 2 pixels and a step size of 1 pixel are used, while in the remaining convolutional layers, a fill size of 1 pixel and a span size of 1 pixel are used. In addition, each residual convolutional layer, except the last two, has a filter size of 3 × 3 and generates 384 feature maps of size 22 × 22. For the penultimate convolutional layer, 256 feature maps of size 22 × 22 are generated using a filter of size 3 × 3. The last convolutional layer, by using a filter of size 3 × 3, generates 1 feature map of size 44 × 44. After the first convolutional layer and the third convolutional layer, there are two max-pooling layers with a window size of 3 × 3, respectively. These two pooling layers have a step size of 2 pixels. The padding size of 1 pixel is used for the first pooling layer only. In addition, a function parameter rectified linear unit (PReLu) [21] is used as an activation function whose parameters can be learned adaptively. It can be described as follows:

(1) $$\begin{array}{c} f\left(x\right)=\max\;\left(0,x\right)\text{.} \end{array}$$

The local response normalization scheme is also applied after each of the ReLu operations. After the output of the second fully connected layer, a softmax layer is used to generate a distribution over the 2 class labels by minimizing the cross-entropy loss between the predicted labels and ground truth labels.

### 2.5. Training Cascade CNN Architecture

The whole process of the cascaded CNN designed in this study is shown in Figure 2. Mainly, the extensive nodal variability is captured from the input 2D ultrasound images by extracting multiple nodal image blocks from thyroid nodules and normal thyroid images (i.e., cropped image patches of size 353 × 353 randomly sampled from these thyroid nodules and normal thyroid images are the input to CNN15). The segmentation probability maps of thyroid nodules and normal thyroid are used as the output of CNN15, and the resulting image patches are then fed into the network simultaneously to compute the recognition features (i.e., the thyroid nodule segmentation problem is treated as a block classification task, ignoring the relationship between image patches). The CNN in this method uses image blocks of normal thyroid and thyroid nodule images as input, then generates segmentation probability maps as output, and uses a multiview strategy to improve the performance of the CNN15-based model. Finally, the CNN4 is trained with random initialization parameters using the plaque data extracted from the thyroid nodule and normal thyroid images. Specifically, image plaques of 64 × 64 size are randomly sampled. The data obtained from these thyroid images are the input to CNN4, which is centered in the corresponding connected region of the segmented probability map generated by segmentation and which occupies 80% of the area of its corresponding connected region in the segmented probability map after segmentation. In addition, the correctly segmented thyroid nodule region is considered as a positive sample, while the other regions are considered as negative samples.

In this study, all parameters of the two CNNs are set as follows: for CNN15, the learning rate is set to 2 × 10^−4^; the parameters *k*, *n*, *α*, and *β* of the local response normalization scheme are set as follows: *k* = 96, *n* = 24, *α* = 0.0005, and *β* = 0.75, and the batch size is 64; in the second normalization layer, *k* = 256, *n* = 16, *α* = 0.0005, *β* = 0.75, and batch size of 64. In addition to this, the initial value of the slope coefficient of the negative part of the control PReLu is set to 0.9 and decreases at a rate of 0.01. For CNN4, the rate is set to 1.0; when epoch exceeds 10, set the rate to 2 to the (epoch - 6/8) power, and the parameters of this local response normalization scheme are set as follows: *k* = 64, *n* = 24, *α* = 0.0005, and *β* = 0.75, and batch size of 64 in the first normalization layer; *k* = 64, *n* = 16, *α* = 0.0005, and *β* = 0.75, and the batch size is 64. Other parameters of CNN15 and CNN4 are set as follows: the standard deviation of random initial weights is 0.01, and the decay of weights is 0.0005; the momentum of weights and deviations are linear at 0.9 within 10 epochs. Also, by minimizing the validation set, we obtained a rough approximation of the best epoch, and all the above parameters and epochs were used to test our CNN-based model on the test set.

## 3. Results and Discussion

### 3.1. Deep Learning Network Model Implementation

CNNs, as a feed-forward neural network, contain three main operations: convolution, rectified linear units (ReLu), and pooling [22, 23]. The neurons in the network can respond to the surrounding neurons and perform digital image processing to accomplish tasks such as target detection, classification, and segmentation [24, 25]. In this study, the raw data are first preprocessed, and then, the model is trained by the migration learning method, and the results are compared.

### 3.2. Image Preprocessing

#### 3.2.1. Digital Image Processing

The redundant images without region of interest (ROI) were removed from the original data. Since there are objective differences in image size, resolution, signal-to-noise ratio, etc., between ultrasound examiners of different manufacturers, it is necessary to first filter the ultrasound image data for its characteristics, mainly using speckle reduction anisotropic diffusion (SRAD) to reduce the amplitude of high-frequency components and prevent the high-frequency band of the speckle reduction anisotropic diffusion (SRAD) filter is used to reduce the amplitude of high-frequency components and prevent the feature information in the high-frequency band from being masked by noise, thus reducing the impact of noise on image quality and model training results. The data in the dataset are grayscale transformed using histogram equalization (HEE). This is then combined with morphological processing to remove the information annotated by the physician during the examination to obtain subimages reflecting the ultrasound image information of the thyroid tissue [26, 27]. The above digital image processing steps make the image features more significant, thus reducing the influence of irrelevant information on the training results.

#### 3.2.2. Data Enhancement

CNNs' models require a large amount of data as support for training the network, but it is difficult to find sufficient data in practice for the project. Insufficient amount of data can make CNNs become overly strict in order to get the consistency assumption, and thus, overfitting phenomenon occurs. Since the output image size of ultrasound examiners of different manufacturers' models and versions vary, the image is randomly cropped to 230 × 230 pixels by using random cropping, which can enhance 1 ultrasound data image several hundred times. However, the actual effect is poor due to the high similarity of the meaningful part containing the thyroid gland. Meanwhile, the training sample size is expanded with the help of other data enhancement methods, mainly of the spatial geometric transformation class, including operations such as inversion, random cropping, random rotation, and random scaling and deformation, which perform affine transformation on the image. The images are filled by an interpolation method to keep the image size consistent. Meanwhile, it has been shown that the data enhancement multiplier should not be too large; otherwise, it will lead to too much redundant data, and the model cannot learn more features from the redundant data and increase the training volume in vain. In this study, the enhancement multiplier is 10, i.e., one copy of data is augmented with nine parallel thyroid ultrasound images to improve the accuracy and generalization performance of the model and avoid overfitting. Finally, the ImageFolder module is used to convert the images into a tensor for computing.

#### 3.2.3. Image Enhancement

In this study, we mainly use the flexible morphology-based white tophat transform method to achieve the enhancement effect on medical ultrasound images.

*(1) Extraction of Feature Values.* Local contrast enhancement is the most useful method to enhance the effective information of an image. According to the feature that the white tophat transform of flexible morphology can effectively extract the bright features in grayscale images, this study first uses the bright feature values of grayscale images extracted by flexible white tophat transform with different structural elements; then, the *i*th layer feature can be expressed as

(2) $$\begin{array}{c} {f_{swth}}^{i}\left(x,y\right)=f\left(x,y\right)-f\left(x,y\right)\cdot \left[B_{i},A_{i},k_{i}\right]\text{,} \end{array}$$

where *f*_*swth*_^*i*^(*x*, *y*) is the gray value of the (*x*, *y*) position of the *i*th feature layer and [*B*_*i*_, *A*_*i*_, *k*_*i*_] represents different structural elements. In this study, *i* = 3, that is, three different structural elements are used, namely, 3 × 3, 5 × 5, and 7 × 7 shapes (but the middle cross is 1, and the remaining positions are 0) to propose 3 layers of bright eigenvalues.  Figure 3 shows the original image and the eigenvalues of each layer.

In Figure 3, we extract bright eigenvalues through the white tophat transformation of flexible morphology. It can be clearly seen that the larger the template is, the more eigenvalues are extracted, and the noise is also extracted accordingly.

*(2) Enhanced Algorithm.* In order to suppress the enhancement of noise and greatly enhance the brightness of the edge, this algorithm selectively enhances the brightness of the edge to ensure that the noise is not enhanced. We set a threshold *m*, try to ensure that the point (*x*, *y*) where the gray value greater than *m* is located is the edge part, and the point where the gray value less than *m* is located is the noise part or the uniform tissue, and then, the point greater than the thresholded points is superimposed on the extracted bright feature values of each layer, thereby suppressing noise and enhancing edges and improving the readability of useful information in ultrasound images.

The expression of the augmentation algorithm is as follows:

(3) $$\begin{array}{c} f^{\prime }\left(x,y\right)=\left\{\begin{array}{c} f\left(x,y\right)+\overset{n}{\underset{i=1}{\sum }}k_{i}{f_{swth}}^{i}\left(x,y\right)f\left(x,y\right)\geq m,\\ f\left(x,y\right)f\left(x,y\right)<m\text{,} \end{array}\right. \end{array}$$

where *f*′(*x*, *y*) is the result of the final processing, *f*(*x*, *y*) is the original ultrasound image to be processed, and *f*_*swth*_^*i*^(*x*, *y*) is the grayscale value of the *i*th feature layer (*x*, *y*) position extracted using different structural elements [*B*_*i*_, *A*_*i*_, *k*_*i*_], where *k*_*i*_ corresponds to different values of *k* in the flexible morphological transformation. The use of additive operations in the enhancement algorithm and the avoidance of multiplicative operations can make the intensity of the undercontrast region magnified by a larger multiple than that of the normal one, thus ensuring an effective local contrast enhancement and avoiding the grayscale values of other regions to be overboosted. It is possible that the contrast under-region features are contained in various feature layers of different size structures, and if each layer contains the smallest size feature, then the smaller the size feature the more it is amplified. However, noise is usually isolated and differs a lot from the neighboring gray level, so it also tends to amplify the noise. Therefore, if the amplification of each size feature is to be as equal as possible, the morphological open operation is considered to be idempotent, and after performing the open operation, the image no longer contains peaks smaller than the size of that structure element. Therefore, when finding the structural features of larger structural sizes, it is necessary to solve the tophat transform of the image after the open operation.

*(3) Experimental Results and Simulation*. In this study, a series of medical ultrasound images are used to verify the effectiveness of the proposed flexible morphology algorithm for noise suppression and local contrast enhancement methods in ultrasound images, and the results of its experimental simulation are shown in Figure 4.

The structural elements used in this study are 3 × 3, 5 × 5, and 7 × 7 with the middle cross shape of 1 and the rest positions of 0. A total of 3 layers of feature images are used. In the enhancement algorithm, the threshold *m* is taken to be the two-thirds of the maximum value of gray in the image, namely, =2/3max (*f*(*x*, *y*)). From the experimental results, it can be seen that the algorithm proposed in this secion can effectively enhance the local contrast as well as maintain the image details and improve the readability of the image.

## 4. Transfer Learning

The CNN convolutional neural network model, which has performed well in ImageNet image classification, is selected to iteratively compare and adjust the model parameters through the migration learning method to obtain better classification prediction results. In the field of medical image data, it is difficult to find such a large amount of data. This greatly reduces the difficulty of training the model and saves valuable computing resources and time costs [28].  Figure 5 shows a schematic diagram of migration learning process.

### 4.1. Model Training

As more and more complex architectures are proposed, to ensure better accuracy, the network structure tends to use fewer convolution kernels, such as 1 × 1 and 3 × 3 convolution kernels, which shows that the CNN design should consider computational efficiency. An obvious trend is to adopt a modular structure, which can reduce the design space of our network. Another point is that using a bottleneck layer in a module can reduce the amount of computation, which is also an advantage.

Fixed CNN models were selected to train the network and adjust the network parameters. Three initial CNNs' models of (visual geometry group, VGG) 19, GoogLeNet Inception V3, and dense-convolutional network DenseNet161 were selected, and the network was initialized with pretraining parameters obtained by pretraining on natural image datasets to obtain high-dimensional features of images [29]. The convolutional neural network migration learning process is shown in Figure 6.

### 4.2. VGG 19 Model

The VGG network, developed and built by the Visual Geometry Group team at the University of Oxford, uses several consecutive 3 × 3 convolutional kernels instead of the larger convolutional kernels in the neural network. For a given perceptual field, the use of stacked small convolutional kernels implies more nonlinear layers, which can increase the advantage of the neural network in complex training and can improve the network depth and reduce the parameters while having the same perceptual field, improving the accuracy of the neural network classification to some extent [30].

### 4.3. Inception V3 Model

Google Inception Net innovates structurally by using a global average pooling layer instead of a fully connected layer to reduce the number of parameters and to accelerate the convergence of the neural network during training by introducing batch normalization. The Inception V3 model is a 47-layer neural network model that innovatively splits the two-dimensional convolutional layer into two one-dimensional convolutional layers for the purpose of reducing the training parameters and mitigating the overfitting phenomenon [31].

### 4.4. DenseNet 161 Model

DenseNet can be seen as a special case of the residual neural network ResNet, where the CNNs model of ResNet avoids the problems of gradient disappearance and gradient explosion by establishing short-circuit connections between the preceding and following layers so that the gradients can be propagated backwards during training [32, 33]. The DenseNet 161 model, on the contrary, develops a dense connection that interconnects all layers' mechanism, where each layer takes the parameters of its previous layer as an additional input. The dense convolutional network connectivity mechanism is shown in Figure 7.

For the N-layer network, the DenseNet 161 model contains a total of connections, which is more densely connected than the residual neural network. Moreover, each layer of the DenseNet 161 model directly connects the feature parameters of all its previous layers to achieve feature reuse and improve network efficiency.

The output of conventional CNNs at the *n*th layer is as follows:

(4) $$\begin{array}{c} x_{n}=H_{n}\left(x_{n-1}\right)\text{.} \end{array}$$

ResNet cell: then, at the *n*th layer, the feature function from the previous layer is added as

(5) $$\begin{array}{c} x_{n}=H_{n}\left(x_{n-1}\right)+x_{n-1}\text{.} \end{array}$$

The DenseNet cell then connects all layers before the *n*th layer to do the characteristic function as

(6) $$\begin{array}{c} x_{n}=H_{n}\left(\left[x_{0},x_{1},\cdots x_{n-1}\right]\right)\text{.} \end{array}$$

### 4.5. Model Training Test Analysis

In the classification training, the data were labeled according to the pathological diagnosis result criteria, and the data were randomly divided into two parts, the training set and the test set, according to 75% and 25%, to ensure the objectivity of the classification results and avoid random errors and chance. Considering the GPU, CPU, and memory performance, 150 epochs were chosen to run the 3 models on the same data on the same platform as the reference results. The results are summarized by the highest accuracy in the test set, the average accuracy of 30 epochs after the test set, and the size of the parametric model.

We can see from Table 3 that the final accuracy of the training set of all three models is >98%, where the highest accuracy and average accuracy of the DensenNet 16l model are higher than those of the VGG 19 model and the Inception V3 model, which are 98.27% and 92.95%, respectively, and for the model size, the VGG 19 model is the largest, at 550 MB, while the Inception V3 model and the DensenNet 16l model are closer in size, around 100 MB.

### 4.6. Model Classification Performance Analysis

In this study, CNNs models with pretrained parameters obtained from natural images were trained to extract features and classify ultrasound images of thyroid nodules, while the network parameters were adjusted. Three CNNs models with very different structures and distinctive features, VGG 19 model, Inception V3 model, and DensenNet 16l model, were tested, and better results were trained on all three models, which proved the feasibility of CNNs-based benign and malignant classification of thyroid nodules and laid the foundation for the subsequent research work. The correctness and loss curves of the training set and the correctness and loss curves of the test set for the three models are shown in Figures 8 and 9.

Figures 4 and 5 show that, among the three CNNs models, the VGG 19 model has the fastest convergence speed and the best training effect on the training set, showing good classification performance, but its performance in the test set is inferior to that of the Inception V3 model and the DensenNet 161 model, with an average accuracy of only 88.20%. It is speculated that this is due to the low number of network layers and an insufficient number of hidden layers caused by the unique concise structure of the VGG 19 model, which is insufficient for the extraction of high-dimensional features in the training set, resulting in overfitting of low-dimensional parameters and causing classification bias in the test set [34]. Meanwhile, the VGG 19 model takes up more computational resources and uses more network parameters, almost five times the size of the parameters of the other two network models, so the advantage in training time is not obvious. Most of the parameters in this model originate from the first fully connected layer, and in subsequent tests, it was found that removing part of the fully connected layer has little effect on the network performance, yet it can greatly reduce the network parameters.

The convergence process of both Inception V3 and DensenNet 161 models shows a steady fluctuation upward trend, and the final convergence results are above 98%, with the accuracy of 92.87% and 92.95% on the test set, respectively, which have better classification results. The DenseNet 161 model has an aggressive dense connection mechanism, which has a low number of parameters and a good resistance to overfitting. In general, the complexity of nonlinear functions increases as the depth of the neural network increases. Both Inception V3 and DensenNet 161 models have a final saved parameter model size of about 100 MB, which is a significant advantage over the VGG 19 model. Considering the difference in the number of network layers of each model, the Inception V3 and DensenNet 161 models are more conducive to extracting high-dimensional feature values and are more efficient in training. In addition, due to the unique backpropagation design of the DensenNet 161 model, which requires high video memory, the network architecture needs to be optimized, and a smaller Batch Size needs to be selected during the actual training.

## 5. Model Time Performance Analysis

The results of the temporal performance training of the three models in this study are shown in Table 1. The accuracy and precision of the VGG19, Inception V3, and DenseNet161 models in identifying the pathological images of thyroid nodular lesions were higher than 80%, among which the VGG19 model had the highest recall rate of 84.67%. The DenseNet201 model had the highest recall rate, and AUC and AUC were 84.77% and 0.87, respectively, while the computing time was the shortest at 1986.48 s, and the response time was also the shortest at 16 s, indicating that the model had the best overall performance; the Inception V3 model was the second, and the VGG19 model had the worst recognition ability for pathological images of;thyroid nodular lesions, with a response time 24 times that of the DenseNet161 model, the results are shown in Table 4.

## 6. Integrated Learning Model Performance Evaluation

From the 3 network models trained by migration learning, 2 models are selected two by two to be combined as individual learners for integration. In this study, the image recognition accuracy is the most important observation, and the accuracy is weighted in preference. The results show that the integrated learned models have significantly improved the recognition of pathological images of thyroid nodular lesions compared with the individual models, as shown in Table 5. The Inception V3 integrated model with DenseNet161 had the highest accuracy, precision, recall, and AUC and the best overall performance, followed by VGG19 integrated with DenseNet161. The ROC curves of the integrated learning model for the test set image recognition results are shown in Figure 10, and the confusion matrix is shown in Figure 11. The ROC curves and confusion matrix experimental results also validate the above conclusions.

Model integration learning is the combination of multiple learners to improve the robustness and generalization ability of models to accomplish image recognition, classification, and prediction tasks more efficiently. However, the readability and testability of the model architecture and the way of code generation need to be considered in the model integration process. Based on the individual models, this study performs integration learning to further improve the performance of classification models. As a result of the migration learning phase of the single model, the results of this study show that the model integrated with DenseNet161 by Inception V3 has higher accuracy, recall, and AUC, compared with the single model. In terms of network structure, the residual structure of Inception V3 strengthens the image feature extraction ability of the deep network, and the overfitting resistance and generalization performance of DenseNet161 are very powerful, so the combination of these two networks can complement each other and bring out the overall stronger image recognition ability. In particular, the integrated network is more effective in terms of separate image accuracy, which is most important for pathology diagnosis.

## 7. Discussion

Reproducibility of thyroid nodule and normal tissue detection plays a crucial role in optimal treatment quality and patient prognosis. However, the detection of thyroid nodules in ultrasound images is a challenging problem with uneven appearance, surrounding structures such as veins and lymph nodes, low signal-to-noise ratio, low contrast, and blurred borders. In this study, we use a cascaded CNN-based approach to solve the problem of thyroid nodule detection, which can avoid the potential error caused by inaccurate image preprocessing results and the classification bias caused by a less robust feature set. To the best of our knowledge, although there have been several studies on CAD of medical images based on deep learning, this is the first attempt to detect thyroid nodules using CNNs. The key advantage of CNNs over traditional approaches using manual features designed based on human experience [16–18] is the ability to automatically learn weights and biases to generate data-driven, custom, and task-specific dense feature extractors that maximize the use of the two-dimensional structure of the input image. The parameters of the CNN are tuned by stochastic gradient descent on the agent loss function associated with misclassification errors, and gradients are efficiently computed by a backpropagation algorithm. In our study, the CNN can automatically extract effective features from 2D ultrasound images without any hypothetical characterization of the vision of interest. Different boundaries, different edges, and different multilevel texture features can be automatically learned through different convolutional filtering, pooling, and normalization operations. With good noise tolerance, CNNs can be suitable for handling the intrinsic noise characteristics of ultrasound image data from various ultrasound systems. In addition, within certain limits, CNNs are invariant to geometric transformations, deformations, and illumination.

To evaluate the wide applicability of the proposed method in this study, 22,000 images from different ultrasound systems are studied in experiments with 10-fold cross-validation, which is used to illustrate the effectiveness of the cascaded CNN method. And our method is compared with VggNet, ZeilerNet, PreZeilerNet, and ResNet. The results are shown in Table 6, and Figure 12 shows the FROC curve results for the different CNN models used for detection.

The results in Table 6 show that our method outperforms other CNN architectures in detecting thyroid nodules. In particular, Cascade CNNs have an AUC value of 98.89%, which is higher than other models. On the contrary, the clustering detection results were analyzed at the regional level using FROC analysis. Figure 12 shows that the sensitivity of our method based on Cascade CNNs is the best for the same false positive rate per image. The multiview strategy is used to improve the performance of cascaded CNNs. In addition, our special segmentation method can effectively separate different connected regions so that CNN4 can accurately obtain positive and negative sample methods based on the automatic labels generated by the segmentation. In summary, the Cascade CNNs' method is statistically significant for the detection of thyroid nodules.

However, there are no analytical methods to determine hyperparameters in CNNs (e.g., number of layers and cells and size of filters), and they are mainly obtained empirically, as we performed in this study. Our cascaded CNN could not accurately detect some small nodules from thyroid images (with multiple nodules or complex and similar backgrounds). This is because the large image patches and deep structures we used in CNN15 are not conducive to learning effective features of small thyroid nodules. Some thyroid nodules with complex backgrounds are also not accurately detected due to the similar appearance of thyroid nodules, blood vessels, adipose tissue, etc. More advanced features learned by deep CNN are not accurate.

Meanwhile, this study has the following limitations:

1. limited by the number of pathological sections, which may still lead to model overfitting phenomenon.
2. The training data and validation data of the model are from the First Affiliated Hospital of Lanzhou University, China, and there is a lack of multicenter sample data for external validation of the model performance.
3. There is no analytical method to determine the hyperparameters (e.g., number of layers and cells and size of filters) in CNNs, and they are mainly obtained empirically, as we have conducted in this study. In addition, our cascaded CNN could not accurately detect some small nodules (with multiple nodules or complex and similar backgrounds) from the thyroid images. This is because the large image patches and deep structure we used in CNN15 are not conducive to learning effective features of small thyroid nodules. Some thyroid nodules with complex backgrounds are also not accurately detected due to the similar appearance of thyroid nodules, blood vessels, and adipose tissue.

## 8. Conclusion

Accurate detection of thyroid nodules from two-dimensional ultrasound images is very helpful for thyroid ultrasound interpretation and can improve ultrasound-guided diagnostic performance. In this study, a model based on cascaded CNNs is proposed to detect thyroid nodules, which does not require any prior assumptions on the associated visual features. In this study, we tested three CNNs' models with different network depths, widths, and functions for classification training, and showed that the CNNs models can better extract and classify features of ultrasound images of thyroid nodules, and their results show that the Inception V3 model has similar classification accuracy as the DenseNet 161 model and has a smaller number of parameters, a simpler model, and better robustness. In contrast, the network structure of the DenseNet 161 model is better for training generalization of neural networks with a small sample size, but requires higher hardware requirements; the Inception V3 model is slightly inferior, but runs faster. This research result can assist doctors' diagnosis, reduce their workload, and provide a comprehensive reference basis for clinical diagnosis and treatment. Integrating InceptionV3 and DenseNet161 for learning can improve the recognition of pathological images by a single model. The performance of the cascaded CNNs proposed in this study is significantly improved compared with other methods, and the multiview strategy can improve the performance of cascaded CNNs.

There are no studies focused on the use of this method to detect thyroid nodules. Furthermore, we compared the performance of our method with that of other learning methods. The results show that our proposed model performs significantly better than these methods on ultrasound thyroid nodule images, demonstrating its potential clinical application. This technique can provide physicians with an objective second opinion and reduce their heavy workload to avoid misdiagnosis due to overwork. We recognize that our dataset is not sufficient for deep CNNs to learn advanced features and obtain higher accuracy. Therefore, the actual performance level and more robustness of this scheme need to be further tested in future studies. In addition, we will explore other CNN-based models, such as inputting CNN cascades of different image patches and using separate structures for large and small thyroid nodules, as well as cascading with other methods, to achieve more accurate automatic detection of thyroid nodules.

This study reconfirms that artificial intelligence has greater advantages and better application potential in pathological image recognition, and we will subsequently work on improving the accuracy of pathological image recognition of thyroid nodular lesions, improving model performance, establishing a database of thyroid nodular lesion images, and promoting the clinical implementation of the corresponding research results to truly serve the clinic and benefit the majority of patients.

## Figures and Tables

**Figure 1:** Detailed structure of CNNs. Conv: convolutional layer; MP: max-pooling layer; Fc: fully connected layer; DS: double size layer.

**Figure 2:** Flowchart of image block classification based on the cascaded CNN model proposed in this study.

**Figure 3:** Bright feature renderings extracted from different templates. (a) Original images. (b) 3 × 3. (c) 5 × 5. (d) 7 × 7.

**Figure 4:** Flexible morphology enhancement effect diagram. (a) Original image. (b) Enhanced algorithm. (c) Original image. (d) Enhanced algorithm.

**Figure 5:** Schematic diagram of the transfer learning process.

**Figure 6:** Flowchart of migration learning of CNNs.

**Figure 7:** Schematic diagram of the connection mechanism of dense convolutional network.

**Figure 8:** Correctness and loss curves of the training set for the three models.

**Figure 9:** Correctness and loss curves of the test set for the three models.

**Figure 10:** Subjects' operating characteristics profile of the effect of integrated learning model on the test set image recognition.

**Figure 11:** Confusion matrix of the effect of integrated learning model on image recognition of the test set.

**Figure 12:** FROC curves based on the cascaded CNN and other different methods.

**Table 1:** Structure of CNN15 used in this study.

Layer	Input	Filter	Padding	Stride	Output
Conv1	353 × 353, 2	13 × 13, 96	6 × 6	2 × 2	177 × 177, 96
Max-pooling1	177 × 177, 96	3 × 3	1 × 1	2 × 2	89 × 89, 96
Conv2a	89 × 89, 96	5 × 5, 256	2 × 2	2 × 2	45 × 45, 256
Conv2b	45 × 45, 256	5 × 5, 256	2 × 2	1 × 1	45 × 45, 256
Max-pooling2	45 × 45, 256	3 × 3	0 × 0	2 × 2	22 × 22, 256
Conv3	22 × 22, 256	3 × 3, 384	1 × 1	1 × 1	22 × 22, 384
Conv4	22 × 22, 384	3 × 3, 384	1 × 1	1 × 1	22 × 22, 384
Conv5a	22 × 22, 384	3 × 3, 384	1 × 1	1 × 1	22 × 22, 384
Conv5b	22 × 22, 384	3 × 3, 384	1 × 1	1 × 1	22 × 22, 384
Conv5c	22 × 22, 384	3 × 3, 384	1 × 1	1 × 1	22 × 22, 384
Conv5d	22 × 22, 384	3 × 3, 384	1 × 1	1 × 1	22 × 22, 384
Conv5e	22 × 22, 384	3 × 3, 384	1 × 1	1 × 1	22 × 22, 384
Conv5f	22 × 22, 384	3 × 3, 384	1 × 1	1 × 1	22 × 22, 384
Conv5g	22 × 22, 384	3 × 3, 384	1 × 1	1 × 1	22 × 22, 384
Conv5h	22 × 22, 384	3 × 3, 384	1 × 1	1 × 1	22 × 22, 384
Conv5i	22 × 22, 384	3 × 3, 256	1 × 1	1 × 1	22 × 22, 256
DS	22 × 22, 256	—	—	—	44 × 44, 64
Conv6	44 × 44, 64	3 × 3, 1	1 × 1	1 × 1	44 × 44, 1

conv denotes convolutional layer; DS denotes double size layer; the format of the data in the table is size × number.

**Table 2:** Structure of CNN4 used in this study.

Layer	Input	Filter	Padding	Stride	Output
Conv1	64 × 64, 2	5 × 5, 64	2 × 2	1 × 1	64 × 64, 64
Max-pooling1	64 × 64, 64	3 × 3	1 × 1	2 × 2	32 × 32, 64
Conv2	32 × 32, 64	5 × 5, 64	2 × 2	1 × 1	32 × 32, 64
Max-pooling2	32 × 32, 64	3 × 3	1 × 1	2 × 2	16 × 16, 64
Conv3	16 × 16, 64	3 × 3, 64	1 × 1	1 × 1	16 × 16, 64
Max-pooling3	16 × 16, 64	2 × 2	0 × 0	2 × 2	8 × 8, 64
Conv4	8 × 8, 64	3 × 3, 384	1 × 1	1 × 1	8 × 8, 384
Max-pooling4	8 × 8, 384	8 × 8	0 × 0	8 × 8	1 × 1, 384
Fc1	1 × 1, 384	—	—	—	1 × 1, 192
Fc2	1 × 1, 192	—	—	—	1 × 1, 1

conv denotes convolutional layer; Fc denotes fully connected layer; the format of the data in the table is size × number.

**Table 3:** Training test results of three models.

Models	Final accuracy of the training set (%)	Maximum accuracy of the test set (%)	Average accuracy of the test set (%)	Model size(MB)
VGG 19	>98	93.86	88.20	550
Inception V3	>98	98.10	92.87	105
DenseNet 161	>98	98.27	92.95	112

**Table 4:** Evaluation indexes of the temporal performance of the 3 models on the test set images.

Model	Operation time (s)	Recall rate (%)	Response time (s)	AUC
VGG19	2147.58	80.67	389	0.85
Inception V3	2087.31	83.67	40	0.65
DenseNet161	1986.48	84.77	16	0.87

**Table 5:** Evaluation indexes of the effect of the integrated model on test set image recognition.

Model	Accuracy (%)	Precision (%)	Recall rate (%)	AUC
VGG19 + inception V3	83.27	79.46	88.68	0.84
VGG19 + DenseNet161	88.35	85.45	89.52	0.88
Inception V3 + DenseNet161	89.78	87.78	94.57	0.90

**Table 6:** Comparative analysis of AUC performance and 95% confidence interval CI of different models (number format of AUC: mean (standard deviation); *p* < 0.05 is considered to be statistically significant).

Method	AUC (%)	CI (%)	*p* value
CascadeCNNs	98.89 (0.0015)	[97.95 98.96]	2.37*e* − 08
ZeilerNet	94.03 (0.0025)	[93.95 95.42]	7.88*e* − 07
VggNet	92.58 (0.004)	[92.21 93.80]	1.19*e* − 07
ResNet	94.59 (0.0035)	[93.76 94.71]	1.56*e* − 06
PrezeilerNet	94.21 (0.002)	[93.95 95.20]	7.55*e* − 07

## Data Availability

The figures and tables used to support the findings of this study are included within the article.
